# A Model of Social Support for a Patient–Informal Caregiver Dyad

**DOI:** 10.1155/2022/4470366

**Published:** 2022-10-04

**Authors:** Małgorzata Pasek, Lilia Suchocka

**Affiliations:** ^1^Department of Nursing, Faculty of Health, University of Applied Sciences in Tarnów, 33-100 Tarnów, Poland; ^2^Faculty of Education and Psychology, Jan Kochanowski University of Kielce, 25-029 Kielce, Poland

## Abstract

**Background:**

Close persons (informal caregivers) are the most important providers of support indicated by cancer patients. Cancer affects couples as a codependent system. The aim of this study was to investigate the factors influencing the multidimensional aspect of social support in a cancer patient–informal caregiver dyad.

**Methods:**

The research project was cross-sectional. The diagnostic survey method and the survey technique were used. The study was conducted using standardised research tools: BSSS, POS, SSCS, TIPI, ET, SPT, and the authors' own tool for sociodemographic assessment.

**Results:**

Patients and caregivers experienced injustice, exclusion, and a sense of loss with a similar intensity. Statistically significant differences between the examined patients and their caregivers were obtained for the support currently received (*p* < 0.01), emotional support (*p* < 0.05), and the general level of protective buffering support (*p* < 0.001). A higher level of information support for caregivers increases the need for support and a sense of support for patients.

**Conclusion:**

The quality of functioning and mental well-being of patients is directly influenced by the way their caregivers experience the situation of caring for them; negative or positive states of caregivers, affecting the condition of patients, may affect the course of treatment and contribute to or delay the improvement of the state of health. The subjective sense of support in patients during treatment depends on the need for help that is shown to their caregivers. The sense of support variable is subjective and sometimes disproportionate to the support received and given. Therefore, both the patient and their loved one should be provided with care during the treatment process. In the treatment process, both patients and their caregivers need more protective buffering support that allows them to overcome difficulties related to stress, anxiety, and insecurity, thus weakening their negative effects rather than functional support: emotional, information, instrumental, or material.

## 1. Introduction

Cancer is a specific disease which deeply affects a patient's life, engulfing all its spheres and also influencing the closest person. A growing body of research proves that cancer affects couples as a codependent system and that pair-based psychosocial interventions are effective in reducing stress and improving coping skills in a difficult situation [1–4]. In fact, when dealing with cancer, couples may react as an individual, not as individuals [5].

The perceptual definition of social support used in our project has made it possible to highlight important aspects of this concept: the levels of support obtained from various sources and the degree of satisfaction that an individual experiences with this support, as well as the buffering effect of social support on the stress on human mental health [6]. Social support is a moderator and has a positive effect on psychological functioning even after the occurrence of a stressor [7].

Supporting the health of cancer survivors and their families, from diagnosis to survival, is a recognised priority. Promoting the healthy behaviour of cancer survivors in a family context can leverage existing support networks and improve the health of family members performing supportive roles [8]. National institutions also see the need to focus on patient–caregiver dyads in order to improve cancer treatment, as well as to create strategies for integrating caregivers into formal healthcare environments [9].

A better understanding of the challenges faced by cancer-coping couples and a deeper insight into how to broaden coping together can contribute to improving the quality of cancer care [5]. The emotional and informational support offered by caregivers influences patients' activation, which significantly contributes to their conscious participation in the treatment and adherence to the prescribed treatment regimen [10].

Patients diagnosed with cancer have a high level of unmet needs, particularly for psychological support and medical information. Their caregivers also have needs and concerns in relation to the disease. Authors examining couples noted that caregivers should be aware of the health consequences of cancer and consider appropriate supportive care for their loved ones [11].

Early intervention for a patient and their caregiver, and proper social support, may prevent later development of mental stress in both of them [12]. Research by Kelley et al. is concerned about the relationship between social support and health among cancer patients and their caregivers. It showed that social support has a positive effect on patients' and caregivers' perceptions of health at every stage of this neoplastic disease, and the effects can vary depending on the location of the cancer and time. In dyads where patients had lung cancer, 12 months after diagnosis, social support for the patients was correlated with better health conditions reported by their caregivers, and social support for caregivers was correlated with better health conditions reported by the patients. This relationship was not demonstrated in dyads where patients had colorectal cancer [13]. It is important to measure the need for support individually and to provide it properly [14]. A multifaceted analysis of available results allowed Turchi et al. to consider the need to define research protocols and useful management strategies for improving the overall health of cancer patients and those around them. The oncological diagnosis and its repercussions for the lives of patients and their caregivers were examined, and the critical aspects that emerged from the literature were highlighted [15].

Research on the assessment and need for social support in patient–caregiver dyads showed that patients perceived the support received more than caregivers. Detailed characteristics of the caregivers' relationship with patients revealed that caregivers–partners and caregivers–children showed a higher level of perceived support than caregivers–siblings and caregivers–parents. Caregivers received less support from medical personnel than patients did [14]. Regan et al. indicated in their research that, according to the surveyed couples and doctors, social support provided to patients and their caregivers was potentially beneficial, but most couples did not think they needed specific interventions focused on couples [2].

Health behaviours are an important element of the assessment of the quality of life, including social support in a patient–close person dyad. Research conducted among couples, where patients had lung or colorectal cancer, and one or both partners in the dyad smoked cigarettes indicated worse mental health than in nonsmoking dyads. Cigarette smoking had less impact on the assessment of physical health [16]. In contrast, a study of physical activity revealed that a partner providing support to a patient when undertaking physical activity contributed more to the achievement of effects than individual exercises. The most desirable exercises were those done in pairs, and separate exercises were preferred only when the activity data was made available in an application or on a website [17]. The importance of physical activity has been confirmed by a subsequent study showing that interventions to increase physical activity in adult cancer survivors may not be possible without the support of caregivers. The study has shown a statistically significant relationship, with particular emphasis on such aspects as companionship, motivation, and health promotion [9].

The social support provided for a patient–caregiver dyad is important when cancer treatment is successfully completed. A particularly frequent area of research projects is the study of sexual health and intimate relationships after the end of cancer, which confirms a common understanding of the physical and psychological challenges and the need for support [18–22]. Gorman et al. found that both convalescents and their partners revealed a spectrum of ways in which couples deal with changes in their relationships and sexual health, stressing that “open communication” and “teamwork” strategies are critical [23]. Survivors' and caregivers' needs for supportive care and responsibility are interdependent.

Cancer alters the social functioning of a patient–caregiver dyad. This has been confirmed by a study of couples in which women contracted breast cancer. The study distinguished priority factors influencing interactions and relationship requirements. Women prioritised their own needs, sometimes at the expense of their partners and relationships. The relationships were reformulated considering the need for additional support and resources to help the couples maintain their relationships during early survival. It is emphasised that social support should be provided in a timely manner and that targeted resources should be provided [24].

When analysing social support in the context of physical symptoms, attention is drawn to the study by Lambert et al., who noted that caregivers' suffering indicators exceeded not only the population norms but also those reported by the prostate cancer patients themselves. The authors postulated that coping skill interventions should address the affected couple as an individual and increase the ability of both partners to overcome cancer-related challenges [25].

Additional variables were introduced into the research. The meta-analysis by Nissen showed that a high level of insecure attachment affected the low level of social support, but also a higher level of depression and anxiety symptoms in cancer patients and their caregivers [26]. A common understanding of their own needs in the dyad motivates partners to ask for support. Informal and formal social networks are also helpful in providing multidimensional support, which makes it possible to avoid experiences of isolation and helplessness in the face of disease. Psychosocial support has been defined as the basic dimension helping couples maintain a positive relationship in the dyad, in both the acute phase of treatment and the early phase of survival [27].

The aim of our study was to investigate the factors influencing the multidimensional aspect of social support in a cancer patient–informal caregiver dyad. Cancer patients indicate that a close person is the most important support provider [14], followed by nurses and doctors.

## 2. Materials and Methods

The project was approved by the local Bioethics Committee of the Krakow Academy (Resolution No. 29/2015 of 14 May 2015).

### 2.1. Study Assumptions

The study assumptions are shown in Figure 1, which graphically describes the theoretical model of social support in the studied group of patients treated for cancer and their caregivers (dyads). To develop this, we analysed scientific research reports [14, 28–34], talked to various specialists in oncological care, and also used our own many years of experience in working with cancer patients and their loved ones.

The model assumes that the independent control variables affect the sense and type of social support for patients and their caregivers:

- Personality structure as expressed by extroversion, agreeableness, conscientiousness, emotional stability, openness to experience, and global self-esteem
- Experienced emotions illustrated by the scale of experienced social pain (injustice, exclusion, and loss), emotional state (stress, anxiety, depression, anger, and loss), and affect (positive and negative)
- Attitude during the treatment process, manifested by satisfaction and optimism, self-care and self-compassion, and the need for help
- A patient's condition, reflected on the scale of experienced social pain and emotional state

The model assumes that the sense of social support in a patient–caregiver dyad depends on intervening variables, such as gender, age, education, material status, place of residence, attitude to work, type of relationship to the person with cancer, and the fear of developing the disease.

The sense of social support of the surveyed patients and their caregivers is manifested by the control side variables:

- Perceived available support consisting of the variables: perceived emotional support and perceived instrumental support
- The need for support
- Seeking support
- Support currently received consisting of the variables: emotional support, instrumental support, and information support
- Protective buffering support

We assume that the examined variables indicated above may be mediators for social support.

### 2.2. Research Methods

The research project was of a cross-sectional nature. The diagnostic survey method and the survey technique were used. The research was carried out in the chemotherapy and radiotherapy wards of oncology hospitals in Poland: Krakow, Lublin, Kielce, and Tarnów in the years 2016-2019.

Table 1 shows the studied variable types and the research tools used to study them.

A detailed description of the research tools is contained in the article entitled “Model of Social Support for Patients Treated for Cancer” by Pasek et al. [35].

### 2.3. Participants

Couples—dyads—were invited to participate in the study. Each dyad included a cancer patient and their loved one indicated by them. Couples—dyads including an oncological patient and a close person indicated by the patient—were invited to participate in the study. Respondents were selected by the purposive sampling method, where the type and structure of the sample results from the research objectives assumed, and the elements of the sample are objects corresponding to the research objectives. Therefore, the conditions of including and excluding respondents were carefully prepared. The inclusion criteria for patients were consent to participate in the study, the ongoing neoplastic process, radical cancer treatment (radiotherapy, chemotherapy, or combination therapy) in inpatient wards, and the mental state enabling understanding and independent completion of the questionnaires. The criteria for inclusion in the study for caregivers, that is, the persons indicated by the patients, who were engaged in helping them on a daily basis, were consent to participate in the study and the mental state enabling understanding and independent completion of the questionnaires.

Participation in the study was conscious and voluntary. Questionnaires were given to couples. Having completed them, each patient and their loved one put it in one unmarked envelope, after which the envelope was sealed. This ensured that the principle of anonymity was maintained.

Nearly 300 dyads were recruited for the study, of which 203 agreed to participate in it and received questionnaires to complete. Ultimately, 185 patients and 178 caregivers returned completed questionnaires. Having checked the questionnaires for completeness of data, 170 dyads were qualified for the study.

Table 2 shows the sociodemographic characteristics of the experimental groups.

The mean age of female patients was 55.73 years and of male patients 64.46 years. Among informal caregivers, the mean age of women was 50.32 years and of men 55.41 years. Women constituted the vast majority of patients (over 70%) and slightly more than half (55%) of caregivers.

The respondents, both patients and caregivers, were most often married and had secondary education.

### 2.4. Statistical Analysis

The characteristics of the studied groups were based on the statistical analysis of the size of the groups together with the percentage indicator for the total number of respondents. Due to the significant disproportion in the number of respondents in each group and the distribution of results inconsistent with the normal distribution, a comparative analysis of the groups of men and women for the “age” variable was carried out using the nonparametric Mann-Whitney *U* test.

Determinants of social support were searched based on multiple regression analysis, using the progressive stepwise method. An analysis of residual distribution was performed, and outliers (atypical observations) were removed from individual models (regression equations).

The correlation-regression model was used to verify the theoretical assumptions of the work. The structural equation method and path analysis were used to more fully verify the theoretical model [36].

The calculations were made using the Statistica software package (Krakow, Poland).

In order to verify whether the theoretical model fits the data, structural equation modelling (SEM) was performed using the AMOS software.

The verification of the assumption with a multivariate normal distribution indicated that this assumption was not met in the analysed model, and so estimators resistant to breaking the assumption of a multivariate normal distribution were used: MLR, MLM, and MLMV, and the R package (environment) with the RStudio editor was applied.

## 3. Results

Table 3 shows the values of the variable elements of the individual scales and questionnaires for the experimental groups of patients and their caregivers.

Based on the results obtained, it can be concluded that the studied patients were characterised by a statistically significantly lower (*p* ≤ 0.05) extroversion (5.04), agreeableness (5.44), and conscientiousness (5.49) than the surveyed caregivers. The study did not show statistically significant differences for the features of emotional stability and openness. The values of the examined personality traits were lower for patients compared to caregivers.

Both patients and caregivers experienced injustice, exclusion, and a sense of loss at a similar intensity.

Self-care and the need for compassion were shown to a greater degree by caregivers than by patients, but this difference was not statistically significant. Nevertheless, based on the result obtained, it can be concluded that in the treatment process, caregivers need compassion more than the patients for whom they care.

On the positive orientation scale, the surveyed patients showed a lower ability to perceive positive aspects of their lives than their loved ones. Their beliefs about the world and the future were less optimistic than those of informal caregivers. The difference was statistically significant (*p* ≤ 0.05).

The levels of experienced stress, anxiety, depression, anger, and need for help in the studied patients was lower than in their caregivers. However, the difference was not statistically significant.

Perceived emotional support, information support, the need for support, seeking support, and instrumental support were not statistically significantly in the studied patients and their caregivers. The above-mentioned types of support were medium in both groups.

On the support scales, statistically significant differences between the examined patients and their caregivers occurred for the support currently received (*p* ≤ 0.01), emotional support (*p* ≤ 0.05), and the general level of received protective buffering support (*p* ≤ 0.001).

On all support scales, the studied patients undergoing cancer treatment showed a greater need for support than their caregivers.

Table 4 shows the correlations between a caregiver's personality and the types of support for a patient.

Our study showed statistically significant differences on the scales of the support currently received and emotional support. In both cases, the values of support indicated by patients were higher than those pointed out by caregivers. On the protective buffering support scale, the sense of support was statistically significantly higher for the caregivers than for the patients. On the other hand, no statistically significant differences were observed in the groups of patients and their caregivers on the scales of perceived emotional support, perceived information support, the need for support, the sense of support, instrumental support, and information support.

There was a statistically significant correlation between information support in the group of caregivers and the need for support (0.23) and the sense of support (0.16) in the group of patients. A positive correlation was obtained, indicating that the need for support and the sense of support in the patients increased along with growing information support for caregivers.

A statistically significant correlation on the protective buffering support scale (0.25) was present in both groups and reflected in the quality and level of comprehensive protective buffering support in both groups during treatment.

The sense of support scale for the group of patients undergoing cancer treatment statistically significantly depends on the features of extraversion and openness (0.20), emotional stability (0.22), the level of life satisfaction and optimism (0.17), and the need for support (0.27) in caregivers. The correlation obtained is positive, indicating that the higher the openness, hope, optimism, and the need for help, the higher the sense of support in patients.

The scale of protective buffering support in the group of patients statistically significantly correlates with openness (-0.16) and with self-compassion and self-concern (-0.21). The negative correlation obtained shows that if the caregivers are characterised by a lack of openness and low self-care in the treatment process, this negatively affects the level of protective buffering support in patients, thus reducing it. Additionally, the sense of support in the group of patients positively correlated with the scales of injustice (0.18), exclusion (0.16), loss (0.30), and the general sense of exclusion and alienation (0.26). This allows us to conclude that if caregivers experience a sense of injustice, exclusion, loss, and general alienation while caring for their loved ones with cancer, the sense of protective buffering support is lower in the patients for whom they care.

Additionally, protective buffering support in the group of patients positively correlated at a statistically significant level with the scales of anxiety (0.24), depression (0.18), anger (0.20), and need for help (0.30) in the group of caregivers. This confirms that if caregivers experience fear and anxiety related to the disease and treatment of their loved ones and states of low mood and sadness, anger, and irritation and they need help during cancer treatment, the sense of protective buffering support is lower in patients.

### 3.1. Verification of the Research Model of a Patient–Informal Caregiver Dyad

Figure 2 shows the model of social support for a patient–caregiver dyad verified by the conducted study.

The statistical parameters obtained indicate that the model explains well the previously assumed hypothetical theoretical model for the groups of patients and their caregivers: Chi − squared = 68.550 is statistically insignificant, RMSEA = 0.007 is good, and NFI = 0.935, CFI = 0.999, and GFI =0.945 are greater than 0.901 and approach 1, which means that the model is a good fit (Table 5).

## 4. Discussion

In social, psychological, and medical statements, cancer continues to be perceived as a death sentence even though it is possible to make a quick diagnosis of a neoplastic disease in many locations and implement effective treatment and modern anticancer therapies and so on. In our study, this is confirmed by the feeling of injustice, exclusion, and loss experienced on a similar level by both patients and caregivers. Ahluwalia et al. indicate that a neoplastic disease contributes to the disruption of the mutual patient's and caregiver's understanding and sense of harmony, while relationships are an important factor influencing the processes of adaptation to the disease situation [37].

Based on the study and statistical analysis, a well-fitting verified research model of support has been obtained. It concerns the study of social support for cancer patients undergoing cancer treatment and their caregivers. The study of patient–caregiver dyads in terms of social support gives the opportunity to perceive the issues of support during cancer treatment as multidimensional and multifaceted. The research of the literature on the subject highlights the correlation between the higher assessment of the patient's quality of life indicated by patients and social support and openness experienced by their caregivers [38].

The studied patients during cancer treatment were characterised by a tendency to depression (0.70), distance to the need for self-compassion (-0.69), and experienced social pain (0.76). The above dependencies of the variables make it possible to conclude that the subjective specificity of the functioning of the studied patients during treatment may be related to the experienced states of depressed mood and sadness, the control of self-compassion and the need for increased concern, and the tendency to feel loneliness, alienation, and inner helplessness during the treatment process. The presence of negative emotions in the course of neoplastic disease has been confirmed by researchers, who also indicate the possibility of helping cancer patients [30, 39, 40].

The social support experienced by the studied patients during treatment was manifested by the variables: the sense of support (0.81) and the need for support (0.68). The positive nature of the correlations indicates that the surveyed patients showed a high sense of support received with a simultaneous increased need for support. Based on the empirical study, it has been confirmed that cancer patients cannot remain alone during treatment and need people who provide them with support, and the sense of support received is additionally correlated with their caregivers' need for help. Our study results confirm empirically the enormous importance of support in oncological treatment. Takeuchi et al. emphasise that patients and their partners are interdependent as cancer affects their mutual life, both emotionally and practically [41].

The variables characterising patients were positively correlated with those explaining social support (0.11). These results confirm that the more patients experience negative depressive states, fail to cope with the disease and treatment, and feel increased pain and social alienation, the more they need support. A study by Dumrongpanapakorn and Liamputtong showed that social support is a factor that significantly contributes to disease management and treatment in women with breast cancer [28].

The variables describing the characteristics of patients in connection with the support (0.11) that patients perceive during treatment and its specificity explain the aspect of protective buffering support during cancer treatment. The study has proved that both patients and their caregivers need more support during treatment that will protect them from the negative effects of stress and difficulties in coping with it during treatment. There was less need for functional support (that is, emotional, information, instrumental, or material).

The protective buffering support variable was 0.24 in the group of cancer patients, which means that the remaining percentage of the explanatory variables was not included in the study. This can be the subject of further research on social support.

The psychological specificity of the surveyed caregivers who took care of their loved ones with cancer was expressed in the need for help (0.78), stress (0.80), anxiety (0.82), depression (0.73), anger (0.77), and exclusion (0.75), having positive connotations. These results empirically confirm that the examined caregivers are prone to experiencing stress and increased anxiety during care, may experience depressive states and moods, as well as anger in connection with the situation, and feel alienated and excluded. At the same time, they feel a strong need for help. The perceived level of stress is positively correlated to anxiety and has a high value, which proves that experiencing negative stress during treatment is manifested by increased anxiety and fear for the patient's condition. Reducing stress and tensions during care gives caregivers the strength and opportunity to control anxiety and fears.

Caregivers' participation in the treatment process influenced the development of a distance to the need for self-compassion (-0.18) and self-care (-0.31) and an increased sense of support, particularly of a protective buffering nature (0.42). Caregivers' distance to the need for self-compassion affected the quality of support for patients, and caregivers' protective buffering support affected (0.19) patients' protective buffering support.

The variables of the sense of exclusion and alienation in the studied patients were additionally correlated with the scale of social pain, that is, the sense of exclusion and alienation in the group of caregivers. The positive correlation (0.31) obtained is statistically quite high and proves that if caregivers feel lonely, excluded and left on their own, patients in this situation feel similar; namely, they cannot cope with the sense of loneliness and alienation.

The sense of support variable in the group of studied patients was additionally correlated with the need for help in caregivers. The results obtained indicate that the way in which caregivers experience the situation of caring for patients influences the patients' sense of support (0.20), expressed through the sense of support (0.81) and the need for support (0.68).

The study showed that the relationship between patients and their caregivers was statistically quite high (0.51). The correlation between the way the caregivers experienced the disease and the quality of functioning and mental well-being of the patients was empirically confirmed.

Based on the positive correlations obtained between the scales, it can be concluded that how and whether caregivers experience the need for help, increased stress, anxiety, depressive states and moods, anger, alienation, and loneliness affect the functioning of patients in the entire treatment process and their need for help. A high value of the positive correlation (0.39) indicates that if caregivers need help, patients simultaneously show an increased sense of support.

Statistical mediators between the levels of protective buffering support in caregivers and their patients were deficiencies in experiencing self-compassion and self-concern in the group of caregivers. This result is indicated by an increased negative correlation between the scales (-0.31). Another statistical mediator is the overall level of experienced protective buffering support in the group of caregivers. The obtained correlation is positive (0.42) and is at a higher level.

It is worth noting that the self-compassion scale in the group of caregivers is explained by three additional variables (e3) that were not included in the discussed model. The protective buffering support scale in the surveyed caregivers is additionally explained by two additional variables (e3), which were also not included in the discussed model. This is an additional justification for continuing the study of support for patient–caregiver dyads.

The study shows that persons who care for their loved ones during cancer treatment experience negative states such as increased stress, anxiety and fear for the affected person's condition, depression, and anger.

In our study, patients showed a lower ability to perceive positive aspects of their lives than their loved ones (*p* < 0.05). Most likely, this may also be related to personality traits. The level of extraversion and agreeableness was significantly lower in cancer patients than in their caregivers. In practice, patients are withdrawn and unwilling to cooperate with medics. Kroemeke and Sobczyk-Kruszelnicka indicate that typical daily coping and the support received were significantly associated with a higher daily positive affect [42], which additionally strengthens the importance of research on social support in dyads during cancer.

### 4.1. Study Limitations

The research project was of a cross-sectional nature. The possibility of conducting longitudinal research can make it possible to trace the dynamics of changes in the perception of social support.

Taking account of, for example, existential aspects in experiencing a neoplastic could indicate important factors influencing the experience of multidimensional support in both patients and caregivers.

Women constitute the majority of respondents in the groups of both patients and caregivers. It is true that the obtained results of the analysis of the studied patients show that the gender variable differentiates the need for support (NS) between the studied women (*M* = 15.16) and men (*M* = 13.36) at a statistically significant level (*p* < 0.01) [35]. However, in subsequent studies (perhaps they would have to be extended in time), we would strive to obtain nearly equally numerous groups in terms of gender.

## 5. Conclusions

1. The quality of functioning and mental well-being of patients is directly influenced by the way their caregivers experience the situation of caring for them; negative or positive states of caregivers, affecting the condition of patients, may affect the course of treatment and contribute to or delay the improvement of the state of health
2. The subjective sense of support in patients during treatment depends on the need for help that is shown to their caregivers. The sense of support variable is subjective and sometimes disproportionate to the support actually received and given. Therefore, both the patient and their loved one should be provided with care during the treatment process
3. In the treatment process, both patients and their caregivers need more protective buffering support that allows them to overcome difficulties related to stress, anxiety, and insecurity, thus weakening their negative effects rather than functional support: emotional, information, instrumental, or material

## Figures and Tables

**Figure 1:** Theoretical model of social support for a patient–caregiver dyad.

**Figure 2:** Characteristics of the model of social support for a patient–caregiver dyad. Chi^2^ = 68.550, df = 68, *p* = 0.458, Chi^2^/df = 1.008, RMSEA = 0.007. P: patients; C: caregivers.

**Table 1:** Investigated variables and the research tools applied.

Variables	Index		Research method
	Patients	Caregivers	
Main variable			
Social support	Perceived available support (PAS) The need for support (NS) Seeking support (SS) Support currently received (SCR) Protective buffering support (PBS)		Berlin social support scales (BSSS)
Independent (control) side variables			
Types of support	Perceived emotional support (PES) Perceived instrumental support (PIS) Emotional support (EmS) Instrumental support (InsS) Information support (InfS) Satisfaction with support (SwS)		Berlin social support scales (BSSS)
Main independent (control) variables			
Personality structure	Extroversion (E) Agreeableness (A) Conscientiousness (C) Emotional stability (ES) Openness to experience (OE)		Ten-item personality inventory (TIPI)
The patient's condition	The scale of experienced social pain Emotional state		Social pain thermometer (SPT) Emotion thermometer (ET)
Attitude during the treatment process	Attitude of satisfaction and optimism Self-care and self-compassion		Positive orientation scale (POS) State self-compassion scale (SSCS)
Attitude towards the person with cancer in the caring process	Attitude of satisfaction and optimism Self-care and self-compassion The need for support		Positive orientation scale (POS) State self-compassion scale (SSCS)
Experienced emotions	Stress Anxiety Depression Injustice Anger Exclusion Loss		Emotion thermometer (ET) Social pain thermometer (SPT)
Intermediate variables			
	Gender Age Education Financial status Place of residence		Personal questionnaire
	Type of cancer treatment Duration of cancer treatment	Attitude to professional work Degree of kinship to the person with cancer Fear of developing the disease	

**Table 2:** Sociodemographic characteristics of the experimental groups.

Variables	Patients		Caregivers	
	*n* Respondents (*n* = 170)	% Respondents	*n* Respondents (*n* = 170)	% Respondents
Gender				
Female	120	70.59	94	55.29
Male	50	29.41	76	44.71
Age (years)				
19–30	7	4.12	8	4.71
31–39	13	7.65	26	1.29
40–49	24	14.12	39	22.94
50–59	38	22.35	39	22.94
60–69	50	29.41	39	22.94
70–79	30	17.65	17	10.00
80–89	8	4.71	2	1.18
Marital status				
Married	119	70.00	147	86.47
Single	13	7.65	9	5.29
Widowed	27	15.88	5	2.94
Informal relationship	8	4.71	8	4.71
Other	3	1.76	1	0.59
Education				
Primary	9	5.29	4	2.35
Vocational	54	31.76	41	24.12
Secondary	66	38.82	62	36.47
Higher	41	24.12	63	37.06
Financial status				
Full-time job	53	31.18	96	56.47
Part-time job or a civil law contract	10	5.88	15	8.83
Disability pension	35	20.59	13	7.65
Retirement pension	57	33.53	32	18.82
Benefits	5	20.59	2	1.18
Pupil/student	0	0	1	0.59
Does not work	10	24.12	4	2.35
Other	0	0	7	4.12
Place of residence				
City	53	31.18	55	32.35
Town	61	35.88	65	38.24
Village	56	32.94	50	29.41
Degree of kinship to the person with cancer				
Husband/wife			94	55.29
Parent			43	25.29
Sibling			16	9.41
Child			4	2.35
Other			13	7.65

**Table 3:** Characteristics of the groups of patients and caregivers based on the research tools used.

Variables	Patients		Caregivers		Mann-Whitney *U* test	
	*M*	sd	*M*	sd	*Z*	*p*
*Personality structure*						
Extroversion (E)	5.04	1.58	5.49	1.42	-2.71	0.007^∗∗^
Agreeableness (A)	5.44	1.35	5.77	1.17	-2.34	0.019^∗^
Conscientiousness (C)	5.49	1.31	5.82	1.19	-2.36	0.018^∗^
Emotional stability (ES)	4.38	1.52	4.46	1.52	-0.63	0.528
Openness to experience (OE)	4.10	1.17	4.32	1.08	-1.46	0.146
*Social pain thermometer*						
SPT.1 injustice	5.22	2.83	5.21	2.75	-0.04	0.967
SPT.2 exclusion	3.36	3.07	2.68	2.57	1.77	0.077
SPT.3 a sense of loss	5.37	3.03	5.23	3.38	0.40	0.690
SPT.WO global value	13.95	7.65	13.12	7.15	0.91	0.364
*State self-compassion scale*						
(SSCS)	37.43	6.36	38.44	5.46	-2.06	0.040^∗^
*Positive orientation scale*						
(POS)	28.41	5.49	30.02	4.83	-2.67	0.008^∗∗^
*Stress thermometer*						
Stress	5.32	3.05	5.72	3.03	-1.12	0.262
Anxiety	5.71	3.05	5.93	2.99	-0.59	0.552
Depression	3.22	3.13	3.10	2.99	0.03	0.972
Anger	4.27	3.28	4.55	3.41	-0.71	0.476
The need for help	4.72	3.19	4.54	3.40	0.53	0.599
*Social support*						
BSSS.PES	13.92	2.41	13.76	2.33	0.64	0.521
BSSS.PIS	14.05	2.53	13.87	2.53	0.33	0.740
BSSS.NS	12.02	2.14	11.64	2.25	1.52	0.128
BSSS.SoS	14.63	3.53	14.12	3.92	1.29	0.199
BSSS.SCR	3.20	0.36	3.09	0.31	3.95	0.000^∗∗∗^
BSSS.EmS	2.96	0.31	2.89	0.26	2.08	0.038^∗^
BSSS.InsS	3.60	0.56	3.49	0.55	2.42	0.015^∗^
BSSS.InfS	3.44	0.69	3.39	0.71	0.64	0.524
BSSS.PBS	2.82	0.77	3.27	0.62	-5.34	0.000^∗∗∗^

^∗^ *p* ≤ 0.05; ^∗∗^*p* ≤ 0.01; ^∗∗∗^*p* ≤ 0.001.

**Table 4:** A caregiver's personality variables and the types of support for a patient.

Patients	Caregivers															
	E	A	C	ES	OE	SPT.1	SPT.2	SPT.3	SPT.WO	SSCS	POS	Stress	Anxiety	Depression	Anger	Need for help
PES	-0.06	0.06	-0.08	-0.01	-0.05	0.00	-0.04	-0.04	-0.03	-0.02	0.03	-0.10	-0.05	0.08	-0.11	-0.04
InfS	-0.10	0.01	-0.07	-0.04	-0.06	0.02	0.01	-0.02	0.00	-0.07	-0.01	-0.06	-0.03	0.10	-0.08	-0.02
SoS	0.14	-0.01	-0.02	0.11	0.01	0.11	0.04	0.04	0.08	-0.05	0.07	0.02	0.08	0.13	0.09	0.19^∗^
SOS	0.20^∗∗^	-0.04	0.11	0.22^∗∗^	0.05	0.13	-0.07	0.04	0.04	0.02	0.17^∗^	0.14	0.14	0.10	0.10	00.27^∗∗∗^
SCR	-0.09	0.02	0.08	-0.03	0.07	0.04	0.00	-0.04	0.00	0.03	0.07	-0.12	-0.11	0.05	-0.15	-0.07
EmS	0.08	0.02	0.03	-0.02	0.03	0.02	0.03	-0.04	0.00	0.03	0.03	-0.11	-0.10	0.05	-0.09	-0.03
InS	-0.05	-0.01	0.11	-0.07	0.10	0.03	-0.03	-0.05	-0.02	0.01	0.10	-0.12	-0.08	0.02	-0.18^∗^	-0.11
InfS	-0.10	0.05	0.06	0.05	0.05	0.08	0.00	0.03	0.05	0.05	0.08	-0.04	-0.08	0.09	-0.08	-0.02
PBS	-0.05	0.14	0.11	0.11	-0.16^∗^	0.18^∗^	0.16^∗^	0.30^∗∗∗^	0.26^∗∗∗^	-0.21^∗∗^	0.13	0.13	0.24^∗∗^	0.18^∗^	0.20^∗∗^	0.30^∗∗∗^

^∗^ *p* ≤ 0.05; ^∗∗^*p* ≤ 0.01; ^∗∗∗^*p* ≤ 0.001.

**Table 5:** Goodness of fit indices.

Goodness of fit indices		
Tucker-Lewis index	TLI	0.999
Comparative fit index	CFI	0.999
Relative fit index	RFI	0.913
Normed fit index	NFI	0.935
Critical *N*	CN	210
Standardised RMR	SRMR	0.038
Root mean square error of approx. (conf. interval 90%)	RMSEA (LO-HI90)	0.007 (0.000-0.047)
*p* of close fit	PCLOSE	0.969
Goodness of fit index	GFI	0.945
Adjusted goodness of fit index	AGFI	0.915
Default model	AIC	142.550
Saturated model	AIC	210.000
Independence model	AIC	1088.450

## Data Availability

The data presented in this study are available on request from the corresponding author.
